# Experiences of Using Weighted Blankets among Children with ADHD and Sleeping Difficulties

**DOI:** 10.1155/2023/1945290

**Published:** 2023-02-14

**Authors:** Maria Lönn, Katarina Aili, Petra Svedberg, Jens Nygren, Håkan Jarbin, Ingrid Larsson

**Affiliations:** ^1^Department of Health and Care, School of Health and Welfare, Halmstad University, Halmstad, Sweden; ^2^Psychiatry Halland, Region Halland, Halmstad, Sweden; ^3^Department of Health and Sport, School of Health and Welfare, Halmstad University, Halmstad, Sweden; ^4^Department of Child and Adolescent Psychiatry, Region Halland, Halmstad, Sweden; ^5^Faculty of Medicine, Department of Clinical Sciences Lund, Child and Adolescent Psychiatry, Lund University, Lund, Sweden

## Abstract

**Introduction:**

Sleeping difficulties are common in children with attention deficit hyperactivity disorder (ADHD). A sleep intervention with weighted blankets was designed to increase current understanding of using weighted blankets to target children's individual needs in connection with sleep and daytime functioning.

**Aim:**

To explore how children with ADHD and sleeping difficulties experience the use of weighted blankets.

**Methods:**

An explorative qualitative design in which 26 children with ADHD and sleeping difficulties, 6–15 years old, were interviewed about a sleep intervention with weighted blankets. Four categories emerged from qualitative content analysis.

**Results:**

Children's experiences revealed that the use of weighted blankets 1) requires a commitment, by adjusting according to needs and preferences and adapting to the environment; 2) improves emotional regulation by feeling calm and feeling safe; 3) changes sleeping patterns by creating new routines for sleep and improving sleep quality; and 4) promotes everyday participation by promoting daily function and balancing activity and sleep.

**Conclusions:**

Using weighted blankets promoted children's management of daily life with ADHD and sleeping difficulties. Occupational therapists can improve the assessment and delivery of weighted blankets tailored to individual needs based on increased knowledge from the children themselves.

## 1. Introduction

Sleep is necessary for health maintenance [1, 2] and the performance of daily activities [3, 4]. Establishing and maintaining good sleep is an issue for children in general but is particularly challenging for children with attention deficit hyperactivity disorder (ADHD) [5], with 25–50% experiencing sleep problems, particularly during initiation and maintenance of sleep [6–8]. Difficulties in regulating emotions and behavior have been suggested to be associated with children's sleep [9]. This is particularly challenging for children with ADHD, who often experience self-regulation difficulties [10] that affect their health and daytime functioning [11, 12].

Ensuring healthy lifestyles and promoting well-being needs to start early, especially in children with ADHD, who will encounter lifelong challenges in everyday performance and participation. Occupational therapists and other professionals within social welfare and healthcare thus need to both acknowledge the importance of sleep as a core occupational category influencing performance and participation in everyday activities and provide appropriate sleep interventions tailored to individual needs [3, 4, 13].

Existing occupational therapy sleep interventions can generally be divided into interventions that target bodily functions, the environment, and daytime activity focusing on occupational balance [4]. Weighted blankets are an intervention targeting bodily functions and the environment. They are used in healthcare settings for treatment of anxiety and sleep problems [14, 15] as a cognitive assistive technology [16] and a sensory integration-based intervention [17]. The use of weighted blankets has been praxis for several diagnoses and settings, most commonly in ADHD [18, 19]. However, whether weighted blankets should be used within healthcare settings has been up for debate [19–21]. There is a lack of evidence and knowledge about using weighted blankets [15, 22]. In order to deliver evidence-informed assistive technologies, increased professional knowledge is needed where research is based on user experiences [23].

Clinical expertise in the use of weighted blankets is based on deep pressure and sensory integration theory. The deep pressure techniques are noninvasive and easily applied interventions without side effects [24], hypothesized to reduce the physiological level of arousal and stress [24, 25]. Furthermore, sensory integration-based interventions such as weighted blankets assist individuals to more effectively self-regulate their emotional and physiological arousal in response to sensory input [26]. Weighted blankets have a calming effect through sensory pathways, reducing hyperarousal, stress, and anxiety and reducing fear responses through safety signals of deep pressure [27, 28]. Children with ADHD and sleeping difficulties could thus be particularly suitable for this kind of intervention, often experiencing difficulties in the self-regulation of arousal and emotions [10, 29].

The current body of knowledge needs to include children's experiences if weighted blankets are to be available as an assistive technology. Individualized care, typical for assistive technology [22, 23], needs to collect individual experiences from the target group in a systematic manner in order to ensure that the children's view is taken into account. Previous knowledge exploring weighted blankets in children with ADHD has informed the current body of knowledge based on parent interviews [17, 30], parent questionnaires [31], parent sleep diaries [31, 32], and objective sleep measurements [31, 32] and is to the best of our knowledge lacking children's experiences of weighted blankets. We need to be aware of children's experiences in order to improve the delivery of tailored interventions and the prescription of assistive technology [23, 33]. Without listening to children themselves, it is hard to ensure that their needs and preferences are being met. Children have the right to express their views in matters that concern them [34], and interventions delivered to children should thus also take their opinions into account. This study will contribute to an expanded body of knowledge, improved guidelines, and an improved capacity for delivering weighted blankets to children in need of improved sleep and well-being. The aim of this study was thus to explore how children with ADHD and sleeping difficulties experience the use of weighted blankets.

## 2. Materials and Methods

### 2.1. Study Design

This study has an explorative qualitative design with an inductive approach [35, 36]. An inductive approach was chosen due to the lack of previous knowledge of the phenomenon [37]. The study adheres to the Consolidated Criteria for Reporting Qualitative Research 32-item checklist, ensuring its trustworthiness [38].

### 2.2. Setting and Participants

Participants in this study were children who participated in a sleep intervention with weighted blankets, which took place between November 2019 and June 2022 at the ADHD unit at a Child and Adolescent Mental Health Service (CAMHS) [39] in the south of Sweden. The children used both a fiber-weighted blanket (4–10 kg) and a light control blanket (2 kg). Families were instructed to try two different types of fiber blankets as part of a sleep intervention study. The children were later asked to participate in interviews after completing 16 weeks of sleep intervention [40] (Figure 1). No new categories or subcategories emerged after the 18^th^ interview, and to ensure that saturation was met, additional eight interviews were conducted before recruitment was terminated in September 2021 [41]. To capture a wide range of experiences concerning the use of weighted blankets, a purposive sample was used [41] based on a variation in age (6–8, 9–10, 11–12, and 13–15 years old), gender (boys and girls), and ADHD subtype (inattentive and hyperactive/combined subtype) (Table 1). Inclusion criteria were uncomplicated DSM-5 ADHD, i.e., without significant comorbidities, confirmed sleeping difficulties, stable pharmacological treatment or no medication, and use of a weighted blanket during the last eight weeks of the sleep intervention. Sleeping problems were verified at the initial visit at CAMHS by three selected questions from the Children's Sleep Habits Questionnaire [42] concerning sleep initiation, sleep maintenance, and sleep duration. The sleeping difficulty should be considered a problem for the family in order to be eligible for the sleep intervention. From the 637 children who attended the ADHD subunit at CAMHS, 86 never received an ADHD diagnosis, ten were not eligible due to comorbidities, and a further 274 did not experience sleeping difficulties. A total of 267 children remained, of whom 99 accepted to participate.

Parents were contacted by telephone after completing the 16-week intervention period. A total of 50 parents and their children were asked to participate in individual interviews, and of these, 26 children accepted. All of these children were eligible and had chosen the weighted blanket as their favorite blanket. The main reasons for families to decline individual interviews were that the child was unwilling to participate (*n* = 19) or social circumstances or health issues in the family (*n* = 5). The median age among children declining was 9 years and 7 were girls (29%). The participating children were 6–15 years old (median age 10 years), 11 were boys (42%), and 15 were girls (58%), and both inattentive, hyperactive, and combined ADHD subtypes were included. Demographic information is displayed in Table 1.

### 2.3. Data Collection

Individual semistructured interviews with children were carried out between May 2020 and September 2021. Fifteen individual interviews were conducted face-to-face in a quiet room at Halmstad University (May-September 2020) with the parent in the next room. Eleven interviews were conducted through the digital platform Zoom (February 2021-September 2021) with the children in their home environment (due to the COVID-19 pandemic). An interview guide was used as well as customized material: a night and day timeline, speech bubbles with pros and cons about the two types of blankets, and figures of children with various feelings. Questions concerned the children's sleep and the use of the weighted blanket, such as “How do you sleep?”, “What does it feel like when you have sleeping difficulties?”, “How do you experience sleeping with a weighted blanket?”, “What has changed since you began sleeping with a weighted blanket?”. Follow-up questions concerned perceived changes during the evening, night, morning, and day and the pros and cons of the weighted blanket. Questions such as “Can you describe your routine when you are about to go to sleep? Fall asleep? Waking up?”, “How do you feel when it's time to go to sleep?”, “Can you describe how you feel when you lie under the weighted blanket?”, “How does it feel in your body? In your head?”, “What do you think about the weighted blanket?”, “Can you tell me something positive? negative?”. The participants were encouraged to provide more in-depth information by asking them if they could “tell more” or posing questions, such as “what do you mean with that?” or “what do you have in mind when you say . . . ?” The customized material was only used during the face-to-face interviews. The material enabled the children to elaborate and facilitated a comparison of the different blankets. The interview guide was tested in a pilot interview which was not included in the study. No changes were made to the interview guide, although distinctions on covering aspects around both night and day timeline was added to complement the customized material. The interviews were 13–62 minutes (median 39 min) with a total duration of 17 hours and 27 minutes. Interviews were conducted by ML, occupational therapist (19 interviews), KA, physiotherapist (6 interviews), and PS, nurse (1 interview). The interviewers were all female and had previous experience interviewing children and/or adults. ML has experience in prescribing weighted blankets and meeting adults with ADHD within an adult outpatient mental health setting on an everyday basis. As a psychiatric nurse, PS also has experience of meeting adults with ADHD. All interviews were audio-recorded and transcribed verbatim.

### 2.4. Data Analysis

The interviews were analyzed using an inductive qualitative content analysis [35, 36, 41, 43]. Analysis began with reading and rereading all transcripts for an initial understanding of the experiences of using weighted blankets, sections of interest were highlighted, and a summary was made for each child, ensuring the original meaning was retained. The analysis then proceeded with the extraction of meaning units into an Excel file including meaning units, codes, subcategories, and categories in order to organize the data and facilitate the analyzing process without fragmenting the data. The extracted meaning units included children's experiences of using weighted blankets, and the categories were created to answer the study's aim to investigate “how children with ADHD and sleeping difficulties experience the use of weighted blankets.” The meaning units (806 pc) were condensed, sorted, and descriptively coded according to shared meaning and close to the text. These extracted codes were then compared, organized, and grouped by ML and IL based on similarities and differences. The analysis was discussed with the research team on several occasions. The process of going back to quotations, checking, and regrouping continued until stability and consensus were met. Finally, eight subcategories were labeled and synthesized into four manifest categories describing children's experiences: *using the weighted blanket requires commitment, using the weighted blanket improves emotional regulation, using the weighted blanket changes sleeping patterns,* and *using the weighted blanket promotes everyday participation.* Representative quotations from the children were used to illustrate the data in the categories.

### 2.5. Ethical Considerations

Ethical approval was obtained from the Swedish Ethical Review Authority, Sweden (no. 2019-02158), and the study followed the principles outlined in the Declaration of Helsinki [44]. All parents and some children gave informed consent in writing during their initial visit at CAMHS. Parental consent was obtained by telephone once again prior to the scheduling of individual interviews. The children were informed about the voluntary nature of participation and the possibility of withdrawing whenever they wanted. Acting in the best interests of children involves allowing them to participate in research and express their opinions. Children are different from adults, and allowing their participation has thus the potential to benefit many children in the future and is at the same time ethical [45].

## 3. Results

Children's experiences were described as *using the weighted blanket: requires commitment, improves emotional regulation, changes sleeping patterns,* and *promotes everyday participation* (Table 2).

### 3.1. Using the Weighted Blanket Requires Commitment

Using the weighted blanket requires a commitment that depends on the children's ability to adjust to needs and preferences as well as adapting to the environment.

#### 3.1.1. Adjusting to Needs and Preferences

The children described different experiences in the process of committing to using the blanket. Individual differences about sleeping with a weighted blanket for the first time were found as the weighted blanket could be experienced as pleasant, comforting, and calming.

*When I had an ordinary blanket, I could not fall asleep. Because then I did not have the weight. When I received the weighted blanket, which was heavy, then I had the weight against my stomach and it was really nice. (Girl 11 years)*

Others experienced the weighted blanket as too heavy, unpleasant, and giving nightmares.

*It was good in one way, but then I got a lot of pain. It was painful in my back and neck when I'd slept with it for a couple of nights. Sometimes I had to take a break, because I could not use it because it was painful. But otherwise it was better, because I could fall asleep quicker ….Maybe it could be made lighter. Maybe it was too heavy for me. (Girl* 13 *years)*

The negative feelings seemed to disappear when the children got used to the weight of the blanket. This was individual and a prerequisite for continued use of the blanket. Establishing an individual commitment to using the blanket with a pleasant feeling was immediate for some, took a few days for others, while in some cases the child was unable to adjust. A number of children felt after some time that the blanket was too light. Even though the blanket felt heavy in the first couple of days, the children adjusted and got used to the weight and thus expressed a need for a heavier one. The possibility of trying different blankets enabled the children to experience a difference from the characteristics of the blankets and enabled them to find a blanket that suited their needs and preferences. In this process, from their ordinary blanket to the weighted blanket and the lighter control blanket, some children found a preference for the weighted blanket, others found a preference for the lighter control blanket, and others found a preference in their ordinary blanket. This process of trying different blankets was described as fundamental, a way of finding a blanket that matched their needs, needing the weight to feel your body, feeling relaxed and embraced, or needing the lighter blanket to be able to move around without pain. Different aspects were expressed and highlighted where the children made adjustments in accordance with their sensory needs in order to improve their sleep. The children described different strategies in this process such as combining the blanket with their ordinary blanket, with pillows or stuffed animals.

*I want both because I have discovered this, that I have the fluffy blanket on first and then the weighted blanket on top. And I usually have my stuffed animal that I have in my hand….and it's fluffy and it has balls in it which are hard, like the weighted blanket. (Girl* 8 *years)*

#### 3.1.2. Adapting to the Environment

Contextual differences affected the children's ability to use the weighted blanket and were a condition for creating an individual commitment and long-term use. Some children experienced difficulties moving the blanket between different households or when going on holiday or having sleepovers. The children rarely considered this as an issue and described how they adapted to the situation finding new and different solutions. Mixed responses were described where the children could be left powerless or on the other hand empowered depending on whether they could adapt to the situation.

*It's very easy to carry. I just take it over my shoulder and walk to the car with my dad. (Girl* 11 *years)*

Being able to manage the weighted blanket in their home context was a precondition for a positive experience of using it and developing an individual commitment. Sleep-related activities such as making the bed, changing sheets, and adjusting the blanket while sleeping were described by the children. The child's ability to manage and use the blanket was dependent of the size and design of the bed, the weight of the blanket, and also on cosleeping parents and siblings. The children described moments of difficulties with managing the blanket in their bed, shifting sleep position and during restlessness, which could result in the blanket sliding of the bed, out of their duvet cover, or too far down in their bed.

*Maybe, it should be a bit lighter…so it does not glide off. I could not lie down against the side of the bed, which I sometimes like doing. Then when I had the weighted blanket, I did that a lot, but I could not do that because I had so little of the blanket left. Like, it slowly glided off the bed and it also pulled my sheets off the bed. It hung down a lot over the edge of the bed. (Boy* 10 *years)*

The children had different experiences concerning seasonal changes and temperature differences. Some children experienced the blanket as too hot, which led to a decreased usage. These experiences were very much contextual, where skylights and summer season were described. Other children experienced positive feelings of the warmth, which was described to decrease restlessness and increase relaxation and feeling of calm.

*I really like it. Because otherwise, I'm not as cold as I usually am. Because when I'm cold I shiver. (Girl* 7 *years)*

The children talked of how their preferences and usage were affected by the opinions of others, where the child adapted to their views. A commitment to using the blanket could thus be encouraged where the child listened to their parents and adapted according to their views.

*Because I actually wanted the light blanket, but mum wanted me to choose the weighted blanket. To help me sleep better. (Boy* 8 *years)*

A question of identity and striving for “normality” without attracting attention was mentioned by one child, who was unable to commit to using the weighted blanket. A commitment to using the weighted blanket was thus described as being dependent on physical as well as social aspects of the environment.

### 3.2. Using the Weighted Blanket Improves Emotional Regulation

The children described how using the weighted blanket could improve their capacity to regulate emotions, creating a feeling of calm and safety when using the weighted blanket.

#### 3.2.1. Feeling Calm

Sleeping with a weighted blanket was experienced as a chance for emotional regulation of arousal, restlessness, impulsive behavior, and anxiety needed in order to fall asleep. The children experienced an increased calmness and less restlessness and thus less need to activate in their routines of trying to fall and stay asleep. Instead of initiating activities such as going to the toilet, drinking water, going to a parent, and using electronic media, the children stayed in bed and fell asleep.

*The blanket stops me from leaving the bed,…Sometimes when I have my ordinary blanket I usually wake up in the middle of the night. And just, wonder what time it is and I get thirsty and stuff like that. Before, I usually went down and had a glass of water, but now with this I usually …Sometimes I get thirsty, anyway, but then I just ignore it and drink in the morning instead. (Girl* 11 *years)*

The children talked of being restless, fiddling, and picking with their things and how they would activate themselves as a strategy to become tired prior to using a weighted blanket, but now they had the blanket instead and felt a calmness enabling improved sleep.

*It's less fiddling now when I have it. Before there was more picking and fiddling. Then I fiddled with things and I was more restless. It may be due to the weight so that I do not move around as much I otherwise do. So maybe I sleep better. (Boy* 12 *years)*

The children experienced being less restless when the blanket stayed in place due to the calming effect of the deep pressure and weight. The children talked of an increased ability to regulate emotions that gave them relief and stimulated better sleep. The children described how the blanket calmed them in the evening when they were full of energy and hyperactive. After a day in school, feeling aroused and unable to calm down the weighted blanket helped them to self-regulate and settle in bed.

*It's like I get calmer and calmer. When I'm calm I get tired more easily. Like today at school, we had a run. We had to do a long run and then I'm not calm at all and later I became really alert. But then when I lay down in my bed and become calmer and calmer, then I can calm down more easily. (Girl* 8 *years)*

#### 3.2.2. Feeling Safe

A comforting, embracing feeling was also experienced, where the weight and pressure were described as creating a sense of security. The weighted blanket was experienced as being a shelter and a place to feel safe in where nothing bad could happen, thus reducing anxiety and promoting better sleep. The children talked of how thoughts of anxiety and fear decreased due to the weight and a new ability to regulate emotions where the child felt safe emerged. Anxiety and fear of something in the dark could occupy the children's minds. A chance to regulate these thoughts increased the child's sense of security, while the weighted blanket gave a safe and comfortable feeling suppressing fears in the dark.

*It feels when you have the light blanket that someone can just pull it off, but with the weighted blanket you feel safer and it's difficult for someone to pull it off…. I do not know whether someone is going to suddenly appear behind the bed and pull the blanket off. But with the weighted blanket, it's more difficult. (Girl* 15 *years)*

### 3.3. Using the Weighted Blanket Changes Sleeping Patterns

A change in sleeping patterns was expressed by the children by creating new routines for sleep and improving sleep quality. The weighted blanket was experienced as an aid to facilitate improved sleep.

#### 3.3.1. Creating New Routines for Sleep

The children experienced how the weighted blanket facilitated a change in sleeping patterns. They described new routines from evening to morning where the weighted blanket became a natural aid enabling the children to fall asleep quicker and manage their daily lives. A change of sleeping patterns with improved routines linked to electronic media and other bedtime activities. They experienced improved routines concerning when they fell asleep and fewer consequences of social jetlag during the transition from the weekend to school nights. The weighted blanket was now described as part of their routine of going to bed, falling asleep, and staying asleep. A change of sleeping patterns was promoted by enhancing the routine, where the addition of the weighted blanket was a cue for sleep, thus improving the children's ability to manage their sleeping difficulty. An improved morning function with new routines was described as a consequence of sleeping through the night, where the child woke up rested and managed their morning routines independently.

*Before I used to be more tired, I usually did not have the energy to get out of bed…My mom usually woke me up, but then I did not have the energy to get up. Yes, I'm really pleased. Now I wake up by myself… and I do that by myself now. I do not have a problem with that. (Boy* 12 *years)*

However, some children spoke of a desire to continue sleeping, staying under their weighted blankets instead of getting on with their morning activities. This was a positive feeling but was also described as having a negative influence on morning routines.

*Sometimes I struggle to get out of bed and sometimes I just want to stay in bed under my warm weighted blanket. It's like both positive and negative, because it's really nice but at the same time I have to struggle to get up and that's really hard. (Girl* 15 *years)*

#### 3.3.2. Improving Sleep Quality

Falling asleep quicker and sleeping through the night was experienced as improving the children's sleep quality, generating relief for the child and the family. The children experienced a change with improved sleep, feeling tired, staying in bed, and sleeping through the night. These changes, which were made discernible for the children by the possibility of trying different blankets, were described in relation to using the lighter blanket and to their ordinary blanket. The weighted blanket was experienced as a new natural aid that was needed to initiate sleep. The strategies they had previously used before participating in the sleep intervention were replaced by the weighted blanket, which was experienced as improving the children's sleep quality.

*It's easier to fall asleep. Because it feels like, you feel like…I cannot explain, but when I do not have a weighted blanket it feels as though I cannot really sleep. (Girl* 13 *years)*

Changes in sleeping patterns when using the weighted blanket improved some of the children's sleep quality, and they felt it took a shorter time to fall asleep and were awakened fewer times during the night. Improved sleep, longer sleep periods, and a deeper sleep were experienced by the children. Although improved sleep was not experienced by all the children, some of the children did not experience a change in their sleep quality. Still experiencing difficulties with sleep initiation and sleep maintenance resulted in a process of going back to sleeping with their ordinary blanket.

*I do not fall asleep at once. I lie awake. (Boy* 11 *years)*

A change in sleeping patterns concerning disturbing thoughts and sounds was described. The children experienced that the weighted blanket helped to promote sleep onset and enhance a deeper sleep. Disturbances due to sensory inputs from their surroundings, such as pets, family members, and outdoor activities, were relieved for some but not for all. The sensory inputs from the surrounding hindered the children to settle down and fall asleep. Being able to ignore sounds with the weighted blanket improved the children's ability to fall asleep and stay asleep.

*I was disturbed by all the noises and then I could not stay still…I do not know what to say. And then I woke up, that really annoyed me as well. Because of that, I did not sleep well. But [with the weighted blanket] it's as though I fall asleep more easily and then when I'm asleep I stay asleep. So I do not get disturbed by the noises anymore and that's really nice. (Boy* 12 *years)*

### 3.4. Using the Weighted Blanket Promotes Everyday Participation

The children experienced that using the weighted blanket promoted everyday participation through improved daily functioning and balanced activity and sleep.

#### 3.4.1. Promoting Daily Functioning

The children experienced a difference in daytime functioning and spoke of changes in attention, mood, and energy. A lesser tendency to withdraw and fewer outbreaks were described as a consequence of an improved mood. Varying experiences with different consequences were described. Some children experienced greater alertness and energy, enabling increased activation and participation in school and leisure activities. Some children described less concentration and less energy prior to using the weighted blanket, where they could fall asleep in class, be less attentive in the classroom, and have low energy levels. Trying different blankets enabled the children to compare and elaborate on conditions and consequences. The children experienced a higher energy level and greater participation in school activities due to increased sleep after having used the weighted blanket.

*It felt bad when I could not sleep, because it was school the next day. So, I could not sleep and I was really tired at school. Now, I get more sleep and I'm more alert during the daytime, so I can work harder at school. (Girl* 11 *years)*

The children described having more energy, which enabled them to get up and become active in the morning, arriving earlier at school and experiencing an improved daily functioning and participation during the day at school as well as in social activities. As a consequence of improved sleep, some children experienced higher attention levels at school, while on the other hand others experienced being less attentive as a consequence of having too much energy.

*I can pay more attention and...It's really nice, because then you get your stuff done, rather than having it left to do…..I go to school, but it's tough. It's hard to string a long and pay attention. You just want to go home and sleep. (Boy* 10 *years)*

Although children could describe experiences of improved sleep, it was sometimes difficult for them to express how having a good sleep could relate to a difference in daytime functioning and everyday participation.

*I do not remember, because it was so long ago I slept with a lighter blanket. So I do not remember, but I think I have slept better now [with the weighted blanket] so I'm more alert. (Girl* 13 *years)*

#### 3.4.2. Balancing Activity and Sleep

The children described improved sleep during the night and more energy during the daytime, which promoted everyday participation. The children experienced less need to sleep in the morning and during the daytime due to their increased energy, thus providing new possibilities for participating in daytime activities. The children described how they did not feel tired during the day and did not have to struggle to stay awake. Instead, they spoke of a new balance with energy during the daytime and tiredness in the evening, promoting participation and better managing daily life with ADHD.

*Now I'm more tired in the evening. I do not have the energy to stay awake that long. Because I'm about to fall asleep with my mobile phone on, then I turn the lights off at once. I'm more tired in the evening, but that's because I've been awake all day. (Girl 13 years)*

While some experienced increased balance due to increased sleep during the night, others experienced an increased balance in their everyday lives due to a new ability to sleep during daytime and an opportunity to recover because of the weighted blanket. The children described how symptoms of headache after a day in school were relieved due to the weighted blanket enabling a more balanced lifestyle and increased participation in everyday activities. Being able to rest, taking a nap and finding new energy and a possibility to be active with friends and leisure activities. One child said:

*You feel rested, and then it's like wakening up and everything is new. Like you have slept a whole night. Because I still sleep deeply even though it's the middle of the day and I can like wake up again and then I'm rested. I mean, I can go out and exercise and such. (Boy* 12 *years)*

## 4. Discussion

Children with ADHD and sleeping difficulties have described their individual experiences of using weighted blankets. According to our results, children committing to the weighted blanket can improve their emotional regulation and change their sleeping patterns. Relieving behavioral and emotional difficulties when trying to fall and stay asleep is described as improving sleep quality and daily functioning in children with ADHD. Taking these aspects into consideration in prescribing weighted blankets may improve their use and outcome in children with sleeping difficulties. The potential of weighted blankets as a self-regulation intervention needs to be acknowledged in order to successfully target the symptoms of children with ADHD and sleeping difficulties.

### 4.1. Using the Weighted Blanket Requires Commitment

The findings showed that being able to manage the weighted blanket independently (in bed and between households) strengthened the children's self-reliance and was a prerequisite for continued use. For example, they needed to adapt to the use of weight. Some children experienced the blanket being too heavy, too light, or becoming lighter over time, thus indicating a need for tailoring the weight to each child. Children have different neurological thresholds for noticing sensory inputs and are thus in need for different strengths of stimuli for optimal outcomes [46]. Adjusting the weight while assessing and closely following up the effects may help to improve commitment to the weighted blanket for each individual child. Children in our study were allowed to change the weight, but only after a request from the parent. A care process where the child has the possibility to share decisions with healthcare professionals could promote the possibilities for continuous use of weighted blankets and the expected benefits of these [18, 19]. The children described different strategies for creating a comfortable feeling when using the weighted blanket. Some of the strategies were dependent on the child's needs and preferences, and some were dependent on contextual variations.

The children described their ability to commit to the weighted blanket as being dependent on parental attitudes, the family situation, the bed environment, and temperature. Some of these contextual factors, for example, light, noise, and temperature, have also been described by healthy adolescents as influential on sleep [47–49]. Aspects in the environment can act as barriers to sleep but also as facilitators of healthy sleep. Strategies for adjustments of the environment can improve sleep, where change of sleeping position, change of light, and temperature have been described as strategies [47, 49]. When stimuli are high, such as noisy family members, hot temperature, and loud music, adjustments may be more difficult [49]. The children's experiences of temperature when using weighted blankets could be due to sensory difficulties [19], their individual thermoregulatory capacity [50], or environmental temperature differences [51, 52]. Comfortable bedding is critical for maintaining sleep [51], and contextual aspects such as the risk of the weighted blanket sliding off the bed and cosleeping family members were also experienced by the children in our study as influencing the use of the blankets. Their use thus needs adjustments that are dependent on both individual and contextual variations. Where some environmental aspects may be resolved by the weighted blanket, other may not and some could be a barrier for continued use. These findings can inform occupational therapists and other healthcare professionals about the importance of delivering weighted blankets tailored to individual needs and preferences of children with ADHD.

### 4.2. Using the Weighted Blanket Improves Emotional Regulation

The children in our study described how the weighted blanket helped them regulate impulsive behaviors, restlessness, arousal, anxiety, and fearfulness. They described having less need of activating themselves at bedtime due to reduced restlessness and anxiety, and instead, they were able to stay in bed and fall asleep. Our findings add new knowledge about how the weighted blanket seemed to create the sense of calm and security that is needed to fall asleep. This is in line with sensory integration theory where sensory interventions are intended to improve attentional, emotional, motoric, communication, and social difficulties. Targeting children's sensory function is proposed as to affect higher level domains in children's motor symptoms and as a consequence also behavioral response [53]. Immediate effects of weighted blankets on mood, behavior, and distress have shown promising results in various daytime settings such as school settings, sensory rooms, hospitals, and dental clinics [54–57]. Research also shows that self-regulation in children is related to adjustment problems and anxiousness and, as a consequence, poor sleep [58]. There is an association between regulation of behavior and emotions and sleep [10, 59], but to the best of our knowledge, research is lacking on its relationship to the use of weighted blankets. Based on our findings, weighted blankets may be an effective sleep intervention as they contributed to improvements in children's behavior and emotions. Using weighted blankets to increase emotional regulation could thus also promote children's sleep; however, more research is needed in this area connecting sensory integration theory, emotional regulation theory, and sleep.

The child's experience of becoming calm and falling asleep when using a weighted blanket is also in line with the theoretical assumptions of social touch, where deep pressure is hypothesized as creating a feeling of calmness, protection, and safety [27, 28]. It is also of interest to discuss this in relation to the sensory regulation theory, by which a behavioral and emotional response is targeted through the child's sensory pathways [53]. The findings from our study add to previous research on the potential of weighted blankets' potential to reduce the core symptoms of children with ADHD [30–32]. Children with ADHD have difficulties in regulating arousal, attention, and behavioral response, and an intervention targeting these difficulties has the potential to improve the symptoms of children with ADHD. However, there is no previous research on how weighted blankets among children with ADHD could improve their ability to process sensory information and regulate emotional responses. Increased knowledge of children's self-regulation ability could improve the delivery of tailored interventions to children with sleeping difficulties and ADHD.

### 4.3. Using the Weighted Blanket Changes Sleeping Patterns

The children in our study experienced improved sleeping patterns such as a shorter time before falling asleep, fewer awakenings, and less disturbance from the environment when using a weighted blanket. Weighted blankets may be an intervention that strengthens the cues of sleep onset by enhancing sensory stimuli in connection to sleep, lowering distraction from other stimuli, and improving the routine connected to preparing/going to sleep [17, 30]. The weighted blankets can help the child to stay in bed, calming down and establish a routine that promotes sleep, and refrain from activating in other activities. This could be especially helpful for children with ADHD with an impaired ability to interpret and inhibit environmental cues connected to sleep onset [60]. Although routines linked to falling asleep and staying asleep are essential for children's sleep patterns, routines linked to waking up are also an issue for children with ADHD and are often neglected in research concerning children's sleeping difficulties [61].

Some children in our study found it easier to wake up in the morning and described greater independence and energy after waking up rested. Others described a desire to stay under the weighted blanket, experiencing difficulties in waking up and leaving the bed. This highlights the complexity of sleep and sleep routines confirming the importance of looking beyond sleep duration [62] and taking a 24-hour perspective when it comes to sleep interventions in children with ADHD. In order to improve routines connected to sleep, the benefits of using weighted blankets may be augmented by combining them with standard sleep hygiene recommendations, which are proposed as constituting part of the first-line treatment for children with ADHD [5, 17, 63, 64]. This is common practice in the prescription process of weighted blankets [19] and will ensure that individual needs are met from evening to morning routines. Children may thus need several different interventions depending on their individual needs [19]. The guidelines for prescribing weighted blankets need to be improved and based on research [15]. This can contribute to ensuring that individual needs are met and that the process of prescribing the blankets is nationally consistent and thus irrespective of regional differences and regulations in healthcare settings.

### 4.4. Using the Weighted Blanket Promotes Everyday Participation

The children in our study have described improved daily functioning, which was confirmed by the parents of the children in a separate study [30]. This is in line with previous research on how improved sleep has the potential to increase children's self-regulation capacity [59] and overall functioning [9, 12, 65]. This thus suggests that increased self-regulation during sleep initiation due to the weighted blanket and increased self-regulation capacity during the daytime due to improved sleep quality have the potential to promote children's overall functioning. Whether these experienced effects are due to the effects of weighted blankets on functioning, as found in a previous study [31], needs further investigation.

The use of weighted blankets both during the day and the night has been described by the children in our study as improving balance and everyday participation in daily activities such as school and leisure activities. When coming home from school feeling exhausted, the weighted blanket was described by a child as an aid that enabled recovery and promoted everyday participation in leisure activities after school. The use of weighted blankets during daytime has been reported previously in individuals with ADHD [17] as well as in other populations as an intervention to decrease anxiety in various daytime settings [15]. From a lifelong perspective and in relation to life imbalance [66], children with ADHD may benefit from interventions in accordance with their individual lifestyles and can manage independently without side effects in their home environment. Improving daily functioning and well-being by an improved ability to balance everyday life is common in occupational therapy practice [67]. However, more research is needed on how children with ADHD can improve their balance between activity and sleep.

### 4.5. Clinical Implications

A clinical implication of delivering individually tailored interventions is the possibility of satisfying the varying needs of different patients and creating a body of knowledge for evidence-based clinical practice with better outcomes, adherence, and cost efficiency [68]. A prescription process for weighted blankets is needed where children are allowed to experience them, and adjustments can be made, and the commitment can be followed up and assessed according to the children's needs, preferences, and contextual barriers. Our results, together with previous and future research, could improve the prescription process for weighted blankets. There is a need for sleep interventions covering different aspects of sleeping [69], and weighted blankets can be one intervention that should be available to meet the diverse circumstances of children with ADHD. By prescribing weighted blankets, occupational therapists can improve children's functioning in relation to sleep as well as to daytime functioning, improve their well-being when trying to fall and stay asleep, and improve their everyday participation as a result of improved sleep. More research is still needed about the effects of weighted blankets. There is a need to acknowledge the individual differences of children in order to deliver successful interventions. By including children in the evaluation of an intervention intended for use by children themselves, we have informed the process of prescribing weighted blankets for children with ADHD.

### 4.6. Methodological Considerations

The trustworthiness of qualitative research can be defined according to the concepts of credibility, dependability, confirmability, and transferability [35].

The *credibility* of our results is strengthened through the rigorous design of this sleep intervention. The children in this study made a choice between a weighted blanket and a lighter control blanket. Only children who chose to use the weighted blanket during the last eight weeks of the sleep intervention were interviewed, ensuring current and long-use experience of sleeping with a weighted blanket. The children were interviewed about their participation in a sleep intervention with weighted blankets without making any preconceived notions of preference. This increases the probability of the children revealing truthful experiences without wanting to please the research team, thus strengthening our findings' credibility. However, a limitation is that we may have missed experiences from children who preferred using the control blanket. Negative experiences of using a weighted blanket could have been revealed to a greater extent in such a sample.

The *dependability* of data is ensured by including a research team with a wide range of perspectives and experiences. ML has previously worked with the assessment and prescription of weighted blankets in a general psychiatric setting that may have biased prior understanding, although a multidisciplinary team has increased the study's dependability. The involvement of two researchers in the analysis process with different preunderstandings also strengthens the dependability, as also the large sample to ensure saturation of the children's experiences. Repeated discussions and cross-checking of data ensured that the categories were grounded in data and did not reflect preconceived perspectives that otherwise could be a threat to the study's trustworthiness. A limitation of the study's dependability may be that the interviews were undertaken by the different coauthors and in different settings. However, this may also be a strength resulting in greater variations in the material.

The *confirmability* was demonstrated throughout the results by including appropriate quotations, rich in quality and content, which ensures that the data correctly represents the children's own experiences. Various experiences were included, with children describing negative as well as positive experiences from using a weighted blanket.

The *transferability* of our results to other contexts is strengthened through a rich description of the participants and setting. Children with ADHD are heterogeneous, and age, sex, and ADHD subtype may affect sleep in different ways [70, 71]. A purposive sample of participants was recruited for diverse perspectives increasing the study's transferability. We have included both boys and girls in our sample, which ensure transferability of our results to both sexes. More boys than girls declined to participate, although we included a large sample size with diverse perspectives from both sexes, which strengthens the study's confirmability. However, the methodology and sample do not allow conclusions being made about girls' and boys' different experiences. A limitation is that all children participated in the same sleep intervention from the same setting, which may be a limitation of transferability to other settings.

## 5. Conclusions

The children experienced that weighted blankets improved their sleep, sleeping patterns, and the balance between activity and sleep but also improved emotional regulation and daily functioning. However, individual needs and barriers to using the weighted blanket may require individual assessment and a close follow-up in order to ensure commitment. A sleep intervention with weighted blankets tailored to individual needs may thus promote children's management of their daily lives with ADHD and sleeping difficulties.

Including children in research and acknowledging the child's perspective is a first step in offering evidence-based clinical guidelines for prescribing weighted blankets. Occupational therapists can improve the assessment and delivery of weighted blankets in order to improve the health and well-being of children with ADHD based on increased knowledge from the children themselves.

## Figures and Tables

**Figure 1:** Study design of sleep intervention with weighted blankets and recruitment of participants for interviews.

**Table 1:** Characteristics of the intervention and participating children with ADHD and sleeping difficulties.

Characteristics of children and intervention	6–8 years (*n* = 6)	9–10 years (*n* = 9)	11–12 years (*n* = 6)	13–15 years (*n* = 5)
Gender				
Boys/girls	3/3	5/4	3/3	0/5
Weight (kg)				
Median, range	27, 19–41	35, 28–42	37, 33–58	45, 43–60
ADHD subtype				
Inattentive/hyperactive/combined	3/2/1	2/0/7	2/1/3	3/0/2
Weight of the blanket (kg)				
6/8/10	6/0/0	5/4/0	4/1/1	4/1/0
Alternates between two households^a^				
Yes/no	0/6	3/6	2/4	1/4

^a^Alternating between households means children with parents living in different households. These children changed households every week. ^b^Sleeping difficulties verified at CAMHS by three selected questions from the Children's Sleep Habits Questionnaire (CSHQ) [42].

**Table 2:** The subcategories and categories describing children's experiences of using weighted blankets.

Children's experiences of using weighted blankets	
Subcategories	Categories
*Adjusting to needs and preferences*	*Using the weighted blanket requires commitment*
*Adapting to the environment*	

*Feeling calm*	*Using the weighted blanket improves emotional regulation*
*Feeling safe*	

*Creating new routines for sleep*	*Using the weighted blanket changes sleeping patterns*
*Improving sleep quality*	

*Promoting daily functioning*	*Using the weighted blanket promotes everyday participation*
*Balancing activity and sleep*	

## Data Availability

Access to raw data is restricted due to ethical considerations.
